# Three in-one fenestrated approaches of yolk-shell, silver-silica nanoparticles: A comparative study of antibacterial, antifungal and anti-cancerous applications

**DOI:** 10.1016/j.heliyon.2023.e18034

**Published:** 2023-07-07

**Authors:** Priyanka Singh, Pranav K. Katkar, Tomasz Walski, Raghvendra A. Bohara

**Affiliations:** a Centre for Interdisciplinary Research, D.Y. Patil Educational Society, Kolhapur, India; b Department of Physics, Sejong University, Seoul, South Korea; c Department of Biomedical Engineering, Wroclaw University of Science and Technology, 50-370, Wroclaw, Poland; d CURAM, SFI Research Centre for Medical Devices, University of Galway, Ireland

**Keywords:** Nanoparticles, Minimum inhibitory concentration, MTT-assay, Prostrate cancer, Energy-dispersive X-ray spectroscopy

## Abstract

Yolk-shell-based silica-coated silver nanoparticles are prominently used in the biomedical field aas well as bare silver nanoparticles for various biological applications. The present work narrates the synthesis and silica coating of metallic silver nanoparticles and investigates their antibacterial, antifungal, and anticancerous activity. Both synthesized nanoparticles were characterized by TEM, and SEM-EDX. The average size of silver nanoparticles was 50 nm, while after coating with silica, the average size of silica-coated silver nanoparticles was 80 nm. The nanoparticles' antibacterial, antifungal, and anticancer properties were comparatively examined *in vitro*. Agar well diffusion method was employed to explore the antibacterial activity against gram-positive bacteria (*Bacillus cereus*) and gram-negative bacteria (*Escherichia coli*) at different concentrations and antifungal activity against *Candida Albicans*. To understand the minimum concentration of both nanoparticles, we employed the minimum inhibitory concentration (MIC) test, against bacterial and fungal strains, which was dose dependent. We learned that bare silver nanoparticles showed high antibacterial activity, whereas silica-coated silver nanoparticles surpassed their antifungal capability over bare silver nanoparticles against *Candida albicans*. The anticancer activity of the as-prepared nanoparticles was executed in opposition to the prostate cancer cell (PC-3) line by MTT assay, which showed meaningful activity. Following this, flow cytometry was also effectuated to learn about the number of apoptotic and necrotic cells. The results of this study demonstrate the dynamic anti-cancerous, antibacterial, and antifungal activities of bare silver nanoparticles and silica-coated silver nanoparticles for a long-lasting period.

## Graphical abstract

Outline showing present work: Fabrication of silver nanoparticles followed by its coating with silica. Detailed anti-cancerous, antibacterial and antifungal studies of both the engineered nanoparticles were brought off. Furthermore, briefly, their comparative studies were also carried out. For the observation of anti-cancerous activities, an MTT assay has been executed. Additionally, the determination of apoptotic cells was found out by flow cytometry. The disc-diffusion method and MIC-assay were performed for antibacterial and antifungal studies.

## 1 Introduction

Science's growing potential to serve in the proximity of molecular scale, atom by atom, merging biological substances and the way of chemistry, physics as well as genetics, and microbiology to invent miniature synthetic substances, is the contribution of bionanotechnology [1]. Advancement in medicine and biotechnology for the detection and treatment of disease relies on accurate knowledge of biochemical and microbiological processes [2,3]. Even though numerous techniques are already available for the diagnosis and treatment of disease; still, this area fascinates the researchers to work on it and find some innovative treatments on the nanoscale [4,5].

In the current era, nanotechnology gained a beam of publicity in medicine because it provides the excellent advantage of the interaction of nanostructures with a body at the scale of molecular level. With the swift development in nanotechnology, the implementation of nanoparticles [6] procured fascination in the biomedical field. Among all the nanoparticles, metallic nanoparticles are acquiring heed for copious applications in nanomedicine. Notwithstanding, hardly a few nano-based products elevated from metal are presently in use for therapeutic purposes [7,8]. Betwixt-and-between, the silver nanoparticle is the most promising product because of its excellent antimicrobial and anti-cancerous properties [9,10]. Silver was accustomed to conserving water since age-old and is considered the cradle of anti-disease resources by Hippocrates. There are proof that to avert the septicemia of the soldier's wound, Egyptians utilized coins made of silver during ancient wars [11,12]. Silver compounds were also used during the First World War against wound infections [13]. After reaching the nanoscale, particles of silver have a miraculous change in physicochemical properties and have exceptional biological activities [14]. The uniqueness of silver nanoparticles broaden their pertinency in antibacterial, antifungal, and anti-cancer therapy [[15], [16], [17]].

Amid numerous kinds of nanoparticles accessible at the current time, nanoparticles having core-shell structures, possess excellent properties, collaborating multiple functionalities into a sole hybrid nanocomposite [18,19]. Assorted patterns of efforts were given to study silver nanoparticles' anti-cancerous, antibacterial and antifungal effectiveness. Still, scant or no attention is given to the comparative study of silver and yolk-shell silver-silica nanoparticles. On that account, the present study was focused on learning about the antifungal, antibacterial, and anti-cancerous effects of chemically synthesized silver nanoparticles and silica-coated silver yolk-shell nanoparticles and evaluating the comparative study of the activity of both nanoparticles. Alteration in silver nanoparticle's functionality with silica gives the nanoparticle idiosyncratic effects because of the biocompatibility, hydrophilicity, and optical transparency along with thermal and chemical stability of the silica; unexpectedly, in aqueous-media also [20,21]. The flexibility of silica in surface moderation as well as in synthesis behavior, offers a distinctive edge to the employment of this material for therapeutic purposes [22,23] because of the applicability in medicine, immune compatibility is a prerequisite condition, that will clinch the non-toxic nature of the material [24,25].

Cancer is a highly complex illness exceptionally unpredictable in its unveiling, evolution, and aftermath. Numerous drugs are available for cancer therapy [26] but most are inefficacious to set foot on-target site in adequate concentrations and systematically deploy the desired pharmacological upshot without triggering irreversible undesired harm to normal cells and tissues [27]. One of the typical sorts of cancer is prostate cancer, which commences whilst prostrate cells evolve anomalously [28]. Though there is historical evidence advising the existence of this cancer since antiquity, the first scientific description of this cancer was brought to notice in 1851 [28]. According to GLOBOCAN 2020, approximately 19.3 million new cases of cancer were reported worldwide, and an estimated 10 million deaths related to cancer happened in 2020. Out of which, 7.3% were because of prostate cancer [29]. There are certain limitations associated with conventional chemotherapeutic drugs [30]. Silver nanoparticles have the potential to avoid various drawbacks of typical therapeutic implementations [31]. Tailor-made silver nanoparticles coated with specific biocompatible nanomaterial can target cancerous cells [32] in a foreseeable manner because these can be specifically intended for expanded drug loading [33], upgraded half-life inside the body, controlled release as well as selective distribution by altering their size [34], composition, surface chemistry, and morphology [35,36]. In the same manner, antimicrobial chemotherapy [34] also demands attention because, lately, resistance to antibiotics by disease-engendering fungus and bacteria has been growing at a breathtaking pace and thus became significant trouble. Bacterial and fungal infections are colossal causes of morbidity and mortality. To overcome this resistance mechanism of pathogenic microbes [22], consideration has been given to silver nanoparticles as an encouraging tool, since it works miraculously on a span of targets in contrast to antibiotics, which have a particular site of execution [37]. Silver nanoparticles showcased magnificent outcomes in detecting and remedying microbial infections by enabling the pick out of target pathogens, reactive and combinatorial freightage of antibiotics, successful antibacterial vaccination, and swift detection of pathogens [38].

The present study also pivots on miraculous antimicrobial activities of silver and silica-coated silver nanoparticles at odds with disease-causing bacterial and fungal strains like - *Escherichia coli* (Gram -ve), *Bacillus cereus* (Gram +ve), and *Candida albicans* simultaneously. We preferred to select *E.* *coli* because it is associated with food poisoning, the uppermost cause of urinary tract infection (75%–95%) [39], seizures, bleeding [40,41], confusion, neonatal meningitis [11], and even kidney failure [37,42,43]. *Bacillus cereus* is also associated with gastrointestinal infection [44] whereas *Candida albicans* infect primarily immunocompromised patients and cause candidiasis named fungal infection [45]. MTT assay exhibits the appreciable anti-cancerous venture of silver and silica-coated silver nanoparticles.

Although these studies have been reported earlier in scientific literature, the comparative study of antibacterial, antifungal, and anticancerous activities of bare silver nanoparticles and yolk-shell, silver-silica nanoparticles have been reported for the first time. Such studies are presented by elaborately employing at least two assays for each application. Comprehensive results recommended a high perspective of both the nanoparticles for application in the biomedical field.

## 2 Experimental

### 2.1 Materials and methods

All the reagents required for synthesising and coating silver nanoparticles were procured from Sigma-Aldrich (USA). Materials used for antimicrobial and anticancerous activity experimentation were bought from HiMedia Laboratories (India). Bacterial strains of *Escherichia coli* (Gram -ve) and *Bacillus cereus* (Gram +ve) were procured from the National Collection of Industrial Microorganisms (NCIM, India). PC-3 cell line was obtained from The National Centre for Cell Science (NCCS, India) an autonomous organization aided by the Department of Biotechnology, Government of India. Aqueous solutions were processed by using sterilized double-distilled water. The reagents/chemicals employed were of analytical grade, so utilized precisely without additional purification.

### 2.2 Synthesis and coating of silver nanoparticles

An altered Turkevich process synthesized bare AgNP (yolk) [25], a chemical reduction route. For this, precisely weighed silver-nitrate (1.5 mM) including double distilled water was incorporated along with tri-sodium citrate by using hot-water bath instrument and followed by stirring, purification, and collection of nanoparticles. To fabricate a shell on AgNP, an altered mode of “Stober” [3] was used. Already synthesized AgNPs were taken in concentrated form and kept for sonication along with ethanol, double distilled water, and ammonia. Thence, tetraethyl orthosilicate (TEOS) was added in droplets under uninterrupted stirring (400 RPM) on a magnetic-stirrer, further whole mixture was incubated overnight at room temperature. After the incubation period, a purification process was carried out. All of the above-mentioned methods are aforementioned in detail in our work [46]. Subsequently, prepared nanoparticles were subjected to spectroscopic and bioactivity studies.

### 2.3 Instrumentation and conditions used for the synthesis

The fundamental composition sizes along with the patterning of the resulting synthesized nanoparticles were examined by utilizing scanning electron microscopy (SEM) and energy-dispersive x-ray spectroscopy (EDX) on Jeol-6360A (Japan) instrument with an operating voltage of 20 kV. For transmission electron microscopy (TEM), we used the Philips CM200 Model type of TEM.

### 2.4 Analysis of antibacterial activity

Agar well diffusion technique was employed to assay the antibacterial and antifungal activity of the prepared silver nanoparticles and silica-coated silver nanoparticles [39,47,48]. For this purpose, two distinct bacterial strains were used, i.e. *Escherichia coli* (Gram -ve) and *Bacillus-cereus* (Gram +ve). The antimicrobial activity of both nanoparticles was calculated compared with the control (ciprofloxacin). The microbial culture of bacterial strain was cultivated on nutrient broth and subsequently dabbed on Petri-dishes consisting of agar media. Three wells were drilled onto the agar facet utilizing an autoclaved well-cutter in each petri plate. Afterward, suspension of both the nanoparticles (1 ml; 0.5 mg/mL) in the first plate and (1 ml; 1 mg/mL) in the second plate were swagged into each of the two wells of the petri-plates and were supplemented with 40 ul of standard drug ciprofloxacin, were supplemented. All the plates were then incubated at 37 °C straight for 24 h. Subsequently, both nanoparticles' antibacterial activities were corroborated by considering the zone of inhibition (in mm) fabricated surrounding the well.

The minimum inhibitory concentration (MIC) assay [49] was also performed to unearth the antimicrobial efficacy of nanoparticles. For this experiment, five various concentrations of nanoparticles were taken (10 μg/mL-50 μg/mL).

### 2.5 Antifungal activity of synthesized nanoparticles

The antifungal action of Ag nanoparticles and Ag@SiO_2_ nanoparticles were investigated by employing Kirby - Bauer agar-well disc diffusion method [40,50]. Stock fungal strain of *Candida albicans* was put together and maintained in media solution. The media for *Candida albicans* was prepared by dissolving Dextrose, peptone, NH_4_H_2_PO_4_, KNO_3_, CaCl_2_ and agar in double-distilled water. The prepared media was then autoclaved at 15 lbs pressure for 15 min at 121 °C. Standard drug Itraconazole was used as a positive control for drug-induced mortality in the antifungal assay. We employed two different concentrations of both nanoparticles to examine their antifungal activities. Similarly, like in antibacterial studies, a minimum inhibitory concentration (MIC) assay was used to demonstrate the antifungal effects of nanoparticles. The colloidal nanoparticles were diluted to acquire the finishing concentration extending from 50 μg/mL to 10 μg/mL and then added to the microtiter plates. Then it was incubated at 37 °C for 24 h. The fungal growth was reckoned by observing absorption (OD) at 600 nm using a microtiter plate.

### 2.6 Cytotoxic effects of Ag and Ag@SiO_2_ nanoparticles

The depletion of tetrazolium salts is extensively acknowledged as a promising route to investigate cell proliferation. The yellow-colored tetrazolium MTT (3-(4,5-dimethylthiazol-2-yl)-2,5-diphenyltetrazolium bromide) is diminished by metabolically dynamic cells, in part by the action of enzyme - dehydrogenase, which produces NADH and NADPH i.e., reducing equivalents. The consecutive intracellular purple formazan can be evaluated by spectrophotometric means. The assay computed the pace by which the cell proliferated, and contrastingly, a metabolic set of events resulted in necrosis or apoptosis.

To analyze the cytotoxic activity of colloidal silver and silica-coated silver nanoparticles, PC-3 cells were trypsinized and added into a centrifuge tube of 5 mL. The prill of cells was procured by vortexing at 300 RPM. The cell count was balanced by using DMEM (Dulbecco's Modified Eagle Medium) media. For every individual well of the 96-well microtiter plate, 200 μl of the cell suspension was supplemented and then the plates were incubated at 37 °C in the atmosphere of 5% CO_2_ for 24 h. Following this, different concentrations (10, 20, 40, 60, 80 μg/mL) of test-sample (nanoparticles) were supplemented to the respective wells and then kept for incubation. After the duration of 24 h, 10% MTT reagent was added, and eventually, it resulted in crystal formation. The solubilization solution (DMSO) was also used to dissolve the developed formazan. Finally, the absorbance was calculated by utilizing a microtiter plate reader at two different wavelengths, i.e., 570 nm and 630 nm. The growth inhibition percentage was evaluated by analyzing the nanoparticle's potency to inhibit the cell growth by 50% (IC50 value).

## 3 Results and discussion

Even though there is an incredible pace of development in the field of nanoscience, relatively very few details are accessible about the upshot of the nanoparticle conjugation process with microbes and with cells and their following consequences. Nowadays, various nanoparticles have been utilized as a drug vector, but their complete synergistic effect inside the human body has not been fully predicted/established. Moreover, there is a requirement for a thorough understanding of nanoparticle-umpired cell death and proper knowledge about the result of this biological phenomenon when the nanoparticle interacts with the cell membrane [51].

The present study was rooted in learning about the antifungal, antibacterial, and anticancerous ventures of chemically synthesized silver nanoparticles and silica-coated silver yolk-shell nanoparticles. Another aspect of the current study was evaluating both nanoparticles' comparative manoeuvre. Silver nanoparticles were synthesized in this work by the chemical-reduction method [25,46], and then uniformly coated by the altered Stober method [20,52]. Both the nanoparticles were characterized decorously by TEM, SEM-EDX. SAED (selected area electron diffraction) pattern of tailored silver nanoparticles, as shown in Fig. 1 (a) depicts a bright randomly dotted ring pattern that describes the crystalline nature of the material because, as we know, the more glaring the spots are, the more crystalline particles will be. Silica-coated silver nanoparticles manifest brighter, thicker, and more continuous rings describing the amorphous coating of silica on the surface of silver nanoparticles, displayed in Fig. 1(b).

**Fig. 1:** Selected Area Electron Diffraction (SAED) pattern of (a) Ag nanoparticles and (b) Ag@SiO_2_ nanoparticles were acquired by administering the electron beam at right angles, perpendicular to the selected domain. Both tailored nanoparticles display concentric rings indicating the nanoparticles' exceedingly crystalline nature. SEM images of the Ag nanoparticles SEM images of the Ag nanoparticles (c), (d), and Ag@SiO_2_ nanoparticles at different magnifications (e) and (f). It is visible that the Ag nanoparticles have a spherical shape and images of Ag@SiO_2_ nanoparticles exhibit a distinct coating of silica layer on the surface of the silver. EDX analysis reveals that prepared Ag nanoparticles contain sodium, chlorine, and some amount of nitrogen and oxygen (g) whereas Ag@SiO_2_ nanoparticles display a burgeoning peak of silica. Some minor peaks of silver, aluminum, sodium, and oxygen are also visible in the represented graph of the elemental analysis (h).

SEM and EDX analyses were carried out to observe the morphology and elemental composition study. It was evident from the SEM analysis, that both nanoparticles were spherical, exhibited in Fig. 1(c)–(f). EDX investigation of the silver nanoparticles confirms the presence of silver in its spectral signal, shown in Fig. 1(g), and (h). Additional elemental tip-offs were also noticed in the spectra which were assigned to the presence of some other compounds.

### 3.1 Antibacterial activity

These days, nanoparticles are very favored among researchers as such materials have astounding nature of killing microorganisms. The benefit of utilizing nanoparticles is the insufficiency of confrontation of microorganisms to their functioning system and glorious application chances. Both the synthesized nanoparticles were highly productive in two conditions as mentioned earlier. Owing to the same reason, the antibacterial effect of silver and silica-coated silver nanoparticles opposed to multi-drug resistant bacteria, challenges and attracts researchers to move forward with this work because of high surface-area to volume proportion and extraordinary physical and chemical qualities. The swift reproduction period of bacteria is among the prominent causes of bacterial infections [53]. Nevertheless, the same reason could be an exemplary strategy to obstruct the possible infection because silver and its related nanoparticles are very fruitful in restraining microbes and have lethal effects on bacteria in a dose and time-dependent fashion [27]. Here, an agar-well technique was employed to appraise the antibacterial activity of both nanoparticles, shown in Fig. 2. Two distinct bacterial strains were taken for this purpose, i.e. *Escherichia coli*(Gram -ve) and *Bacillus cereus* (Gram +ve) [15,54,55]. The nanoparticles were allowed to interact with the bacterial strains in a freshly seeded plate containing medium. 25 mL sterile nutrient-agar was sowed in each of the petri-plate using a glass-rod along with the one-day aged culture of gram +ve and gram -ve bacterial strains distinctly. In each Petri plate, three wells were grooved onto the agar facet using an autoclaved well-cutter. Subsequently, 40 μl of standard drug ciprofloxacin and suspension of both the nanoparticles (1 ml; 0.5 mg/mL) in the first plate and (1 mL; 1 mg/mL) in the second plate protruded into each of the two wells of the petri-plates were seems not natural. Every plate was then incubated at 37 °C straight for one day and night. Eventually, the antibacterial activities of both nanoparticles were validated by calculating the zone of inhibition (in mm) formed around the well (details are given in Table 1, Table 2). It was unearthed from the results, the bacteria that were employed for the experiment died even by using a low concentration of silver as well as silica-coated silver nanoparticles and in a shorter time duration. There is a typical difference between the structure of the cell wall of Gram +ve and Gram -ve bacteria. Gram -ve bacteria possesses a distinguished cytoplasmic membrane, an outer membrane having a weak peptidoglycan layer as well as an external layer containing lipopolysaccharide. In contrast, the cell wall of Gram +ve bacteria possesses a broad peptidoglycan layer accompanying teichoic acid [56]. Because of this difference in the cell wall, nanoparticles (silver and silica-coated silver nanoparticles) behave differently on Gram +ve and Gram - ve bacteria [57]. Although the technique by which nano-scaled silver and its associated nanoparticles work are not entirely known, there are a few possible common mechanisms on which the toxicity of nanoparticles works, as mentioned here [49].

• Both the nanoparticles interact with bacterial proteins by merging the potent effects of thiol (SH) groups, which induces the unnatural, use misfolding of the proteins, and leads to bacterial inactivation [49,58].
• Because of the electrostatic attraction and rapport with sulphur proteins, ions of nanoparticles can cohere with the cell wall and the cytoplasmic - membrane.
• The nanoparticles generate oxidative stress leading to apoptosis-like induced cell death [59].
• DNA and ATP production are interrupted due to the intake of free silver ions [[49], [59]]. As we know, silver nanoparticles regularly release silver ions, which was supposed to be the process of killing microorganisms.

**Fig. 2:** Antibacterial activity of nanoparticles against Gram-positive bacteria *Bacillus cereus* by employing concentrations 1 and 2, (a), (b) respectively. In both studies, Ag nanoparticles manifested vigorous antibacterial activity showing a zone of inhibition of 20 mm, 23 mm, respectively in contrast to silica-coated Ag nanoparticles, with the zone of inhibition of 10 mM and 20 mM (c) antibacterial activities of both the nanoparticles at concentration 1 against Gram-negative bacteria *Escherichia coli*; exhibiting zone of inhibition 17 mM by Ag nanoparticles and 10 mM by silica-coated Ag nanoparticles (d) at concentration 2; Ag nanoparticles revealed zone of inhibition of 10 mM, whereas, silica-coated Ag nanoparticles exhibited 17 mm of inhibiting zone.

The minimum inhibitory concentration (MIC) assay was used to detect the smalles concentration of synthesized nanoparticles against bacterial strain, as shown in Fig. 3(a) & (b). MIC assay has been carried out by repeating the experiment five times, using different nanoparticle concentrations (10 μg/mL- 50 μg/mL). The results obtained from MIC areconsistentt with the disc diffusion results. The lethal effects of both the nanoparticles against bacteria are almost alike or minutely less just in the case of coated nanoparticles.

**Fig. 3:** Minimum inhibitory concentration (MIC) of Ag nanoparticles (denoted in red-colored bars) and Silica coated Ag nanoparticles (shown in black colored bars) against Gram +ve bacteria Bacillus cereus (a). Ag nanoparticles exhibit lofty anti-microbial activity with increasing concentrations whereas coated silver nanoparticles show a lower MIC score. MIC against Gram -ve bacteria - *Escherichia coli* for measuring the activity of Ag nanoparticles and Silica coated Ag nanoparticles (displayed in black -colored bars); both the two nanoparticles revealed higher MIC scores with increasing concentration. The performed experiment showed significant results with a p-value 0.05 in treated concentrations. MIC of Ag nanoparticles and Silica Ag nanoparticles against fungus, *Candida albicans* (c); Ag nanoparticles (denoted in red-colored bars) and Silica coated Ag nanoparticles (shown in black-colored bars). Here coated Ag nanoparticles exhibit towering anti-microbial activity with increasing concentrations, whereas bare silver nanoparticles show a lower MIC score. (For interpretation of the references to color in this figure legend, the reader is referred to the Web version of this article.)

Results are shown here in the Table 1.

**Table 1:** The inhibition zone of Gram -ve bacteria induced by Ag nanoparticles.

*Escherichia coli* (Gram -ve)				
**Sample Name**	**Drug vol.**	**Control** (mean ± SD) [mm]	**AgNPs** (mean ± SD) [mm]	**Ag@SiO**_**2**_**NPs** (mean ± SD) [mm]
**Conc.1(0.5 mg/mL)**		**19 ± 0.50**	**17 ± 1.10**	**10 ± 1.18**
**Conc.2(1 mg/mL)**		**22 ± 1.10**	**20 ± 1.14**	**17 ± 1.20**

**Table 2:** The inhibition zone of Gram +ve bacteria induced by Ag nanoparticles.

*Bacillus cereus* (Gram +ve)				
**Sample Name**	**Drug vol.**	**Control** (mean ± SD) [mm]	**AgNPs** (mean ± SD) [mm]	**Ag@SiO**_**2**_**NPs** (mean ± SD) [mm]
**Conc.1(0.5 mg/mL)**		**23 ± 1.20**	**20 ± 1.30**	**10 ± 1.15**
**Conc.2(1 mg/mL)**		**24 ± 1.20**	**22 ± 2.10**	**21 ± 1.40**

### 3.2 Antifungal

Fungi cause various frantic diseases and remedy of such infection is very necessary because common drugs (amphotericin B, Nystatin, itraconazole, etc) available on market used for treatment cause severe aftereffects such as liver and renal dysfunction [58,60]. Antifungal pursuit of both the nanoparticles was availed by Kirby - Bauer agar-well disc diffusion method (Fig. 4) [50]. We implemented two varied concentrations of Ag nanoparticles and Ag@SiO_2_ nanoparticles to investigate their antifungal activeness. Ag nanoparticles exhibited towering antifungal-action in comparison to Ag@SiO_2_ nanoparticles. The control exhibits 13 mm inhibition zone by using the first and second concentrations respectively (details are given in Table 3). Ag nanoparticles show an inhibition zone of 11 mm when using the first concentration, whereas Ag@SiO_2_ nanoparticles show a 10 mm zone of inhibition. On the other hand, by using the second concentration, Ag nanoparticles, and Ag@SiO_2_ nanoparticles show 9 mm and 12 mm of the zone of inhibition, respectively.

**Fig. 4:** Antifungal activity of nanoparticles against *Candida albicans* by using positive and negative control (a). (b) On concentration 1, both the nanoparticle flaunts approx similar antifungal activities by showing a zone of inhibition of 11 mm (c) On concentration 2, Ag nanoparticles unveil a zone of inhibition of 10 mm whereas silica-coated Ag nanoparticles surpassed antifungal activity over bare silver nanoparticles by exhibiting 12 mm of the inhibiting zone.

**Table 3:** The zone of inhibition of *Candida albicans* induced by Ag nanoparticles.

*Candida albicans*				
**Sample Name**	Drug concentration	**Control** (mean ± SD) [mm]	**AgNPs** (mean ± SD) [mm]	**Ag@SiO**_**2**_**NPs** (mean ± SD) [mm]
**Conc.1(0.5 mg/mL)**		**13.00** **± 1.22**	**11.00** **± 1.18**	**10.00** **± 1.10**
**Conc.2(1 mg/mL)**		**1**.00**± 0.50**	**9.00** **± 1.10**	**12.00** **± 0.50**

The MIC assay of nanoparticles was also evaluated against *Candida albicans* in the range of concentrations form 10 ug/mL to 50 ug/mL (Fig. 3c).

The results showed that with increasing concentrations, the antimicrobial activity of coated Ag nanoparticles is remarkable, while bare silver nanoparticles display a reduced MIC score.

### 3.3 MTT-assay

Currently, one of the most common methods to investigate cell proliferation is the depletion of tetrazolium salts. The viability of PC- 3 cells was calculated by the yellow shaded tetrazolium MTT(3-(4, 5-dimethyl thiazolyl-2)-2, 5-diphenyltetrazolium bromide) colorimetric approach, focussed on the capability of live cells to reduce MTT into formazan crystals. The following intracellular purple formazan can be measured by spectrophotometry. The assay deciphered the rate by which the cell multiplies and numerous metabolic sets of events, as shown in Fig. 5, Fig. 6, Fig. 7, resulting in necrosis or apoptosis. For the MTT assay, the cell density was 10,000 cells. Untreated PC-3 cells were taken as a negative control. The IC_50_ value of the tested nanoparticles for PC-3 cell-line for 24 h of the regimen were calculated and presented in Table 4.

**Fig. 5:** Viability of PC-3 cells after 24 hours of incubation (at 37 C, 5%CO2) with various concentrations of Ag nanoparticles (a) and silica coated Ag nanoparticles in comparison with untreated cells (negative control) and cells treated with cisplatin, evaluated in MTT reduction assay. The IC_50_ value was figured based on the MTT assay of Ag nanoparticles (b) and silica-coated Ag nanoparticles (d).

**Fig. 6:** Optical images of PC-3 cells in control group (a), treated for 24 hours with Ag nanoparticles and silica coated Ag nanoparticles (b) and (c) respectively, revealed significant variations in the morphology.

**Fig. 7:** Microscopic images of the (a) Untreated PC-3 cells and (b) Cisplatin treated PC-3 cells. Changes in the surface structure of the cell-monolayer are observable after treatment with Cisplatin is evident. Morphological variation on the confluency of PC-3 cell monolayer, when exposed to the Ag nanoparticles 10 μg/mL (c) 20 μg/mL (d) 40 μg/mL (e) 60 μg/mL (f) 80 μg/mL (g); for 24 h. The cytotoxic effects of silica coated Ag nanoparticles on PC-3 cell monolayer when exposed to the concentrations: 10 ug/mL (h), 20 ug/mL (i), 40 ug/mL (j), 60 ug/mL (k), 80 ug/mL (l).

**Table 4:** The half maximal inhibitory concentrations of Ag nanoparticles and Silica coated Ag nanoparticles.

Group	PC-3 cell line IC_50_ (in μg/mL) 24h post-treatment
**Cisplatin**	15 μg/mL
**Sample Ag**	37.44 μg/mL
**Ag@SiO**_**2**_	>80 μg/mL (Calculated value: 106.74 μg/mL)

### 3.4 Apoptosis

Apoptosis, a physiological mechanism of cell death, is a promising feature in anti-cancer therapeutic approaches [61]. There are two pathways involved in apoptosis: the extrinsic and intrinsic pathways, both utilizing caspases to execute this physiological process by cleaving a group of proteins [61]. The apoptotic-pathway in cancer is generally inhibited by diversification of overexpression of the protein designated as anti-apoptotic and underexpression of a hallmark of pro-apoptotic proteins [62]. The apoptotic-pathway in cancer is generally inhibited by diversification of overexpression of the protein designated as anti-apoptotic and underexpression of a hallmark of pro-apoptotic proteins [62]. Most of such swapping is the root of intrinsic resistance to the stereotypical anticancer therapy, that is chemotherapy [63,64]. Still, there is a direct need for promising anticancer therapies that will show anticancerous activity by triggering the premeditated cell-death mechanism, i.e. apoptosis [65]. We examined the apoptotic activities of both the synthesized nanoparticles by flow cytometric studies. Typically, the occurrence of the apoptosis is indicated by some distinc morphological features, including loss of plasma membrane asymmetry, bonding and condensation of the nucleus and cytoplasm, and fragmentation of DNA of inter-nucleosome [9]. In the case of apoptotic cells, the phospholipid phosphatidylserine (PS) transitions from the inner space to the outer side of the plasma membrane, resulting in its exposure to the external cellular environment.

Annexin V is a specific Ca^2+^ fostering phospholipid-binding protein with a molecular weight of 35–36 kDa and has high propinquity for PS and interacts with cells to expose PS. Annexin V possibly coalesced with fluorochromes combining fluorescein isothiocyanate (FITC). Since the exposure of PS occurs in the early phase of apoptosis, staining with FITC Annexin V enables the identification of early apoptotic cells compared to assays based upon DNA-fragmentation. The staining of cells using FITC Annexin V allows for detection of membrane integrity loss that initiates the latest phases of cell death which occurs either from necrotic or apoptotic processes, as shown in supplementary file- Figs. 1–3 [66]). So, FITC Annexin V staining is generally employed in combination with a crucial dye, for instance, 7- Amino-Actinomycin Dye (7-AAD) or propidium-iodide (PI) to make it possible for the researchers to recognize early apoptotic cells (Annexin V positive, PI negative). Viable cells with intact membranes exclude PI staining [67].

On the other hand, membranes of injured and dead cells are penetrable to PI. For instance, viable cells are ones, that are PI negative as well as FITC Annexin V negative. PI negative and FITC Annexin V positive cells are in the stage of early apoptosis. In contrast, late apoptotic or hitherto dead cells are positive with PI as well as FITC Annexin V. It is important to mention that described assay does not discriminate between cells gone through apoptotic death or contrarily died owing to necrotic-route because in any case the dead cells are bound to stain [68] with both PI and FITC Annexin V, as shown in Fig. 8. But, if apoptosis is calculated over time, then, cells can be primarily traced from PI and FITC Annexin V negative (that means alive or not quantifiable apoptosis), to positive with FITC Annexin V but negative with PI (early apoptotic, presence of membrane integrity), and finally positive with both - FITC Annexin V as well as PI (that means termination of apoptosis which causes death).

**Fig. 8:** Annexin V - PI expression study of the test compounds, control (a), Ag nanoparticles (b), and silica coated Ag nanoparticles (c) against PC-3 cell line by employing BD FACS Calibur, Cell Quest Pro Software (Version: 6.0).

The observation of cells undergoing all three aforementioned phases indicates apoptosis [69]. However, this singular monitoring approach merely reveals that the cells are positive for both PI and FITC Annexin V. It does not provide comprehensive information regarding the mechanisms underlying cell death. Therefore, there is the need for three-dimensional investigation [70] of cellular models as the majority of current findings regarding apoptosis have been generated using two-dimensional cell culture system [71].

### 3.5 Statistical analysis

All experiments were reiterated five, before analyzing the data and then the demonstrated quantitative data were calculated as means ± standard deviation (SD) ****.

All-inclusive results indicate the emergence of the tremendous potential of silver nanoparticles and silica-coated silver yolk-shell nanoparticles, having exceptionally worthy in the biomedical field.

## 4 Conclusion

In the present work, silver and silica-coated silver yolk-shell nanoparticles were engineered, and further, we mainly emphasized their disease-repelling activities. The prepared nanoparticles were appraised for their antibacterial, antifungal, and anticancer activity. Significant progress has been made in utilizing of engineered silver and related nanoparticles for the treatment of prostrate cancer. Silica-coated silver nanoparticles exhibit a lesser effect compared to bare silver nanoparticles, which can be attributed to the biocompatible nature of silica. In conclusion, our work combines nanotechnology, microbiology, and cancer biology, resulting in the potential development of potent agents with long-lasting effects against cancer, bacteria, and fungi. It is worth noting that both nanoparticles possess these characteristics.

## Author contribution statement

Priyanka Singh: Conceived and designed the experiments; performed the experiments; analyzed and interpreted the data; wrote the paper.

Pranav K. Katkar: Contributed reagents, materials, analysis tools or data.

Tomasz Walski: Analyzed and interpreted the data.

Raghvendra Bohara: Conceived and designed the experiments; analyzed and interpreted the data; contributed reagents, materials, analysis tools or data.

## Data availability statement

Data will be made available on request.

## Declaration of competing interest

The authors declare that they have no known competing financial interests or personal relationships that could have appeared to influence the work reported in this paper.
